# Positively Charged Nanoparticle Delivery of n-Butylidenephthalide Enhances Antitumor Effect in Hepatocellular Carcinoma

**DOI:** 10.1155/2021/8817875

**Published:** 2021-03-19

**Authors:** Kai-Fu Chang, Xiao-Fan Huang, Yu-Ling Lin, Kuang-Wen Liao, Ming-Chang Hsieh, Jinghua Tsai Chang, Nu-Man Tsai

**Affiliations:** ^1^Institute of Medicine, Chung Shan Medical University, Taichung 40201, Taiwan; ^2^Department of Medical Laboratory and Biotechnology, Chung Shan Medical University, Taichung 40201, Taiwan; ^3^Agricultural Biotechnology Research Center, Academia Sinica, Taipei 11529, Taiwan; ^4^Department of Biological Science and Technology, National Chiao Tung University, Hsinchu 30068, Taiwan; ^5^Institute of Molecular Medicine and Bioengineering, National Chiao Tung University, Hsinchu 30068, Taiwan; ^6^Clinical Laboratory, Chung Shan Medical University Hospital, Taichung 40201, Taiwan

## Abstract

Hepatocellular carcinoma (HCC) is the second and sixth leading cause of cancer death in men and woman in 185 countries statistics, respectively. n-Butylidenephthalide (BP) has shown anti-HCC activity, but it also has an unstable structure that decreases its potential antitumor activity. The aim of this study was to investigate the cell uptake, activity protection, and antitumor mechanism of BP encapsulated in the novel liposome LPPC in HCC cells. BP/LPPC exhibited higher cell uptake and cytotoxicity than BP alone, and combined with clinical drug etoposide (VP-16), BP/LPPC showed a synergistic effect against HCC cells. Additionally, BP/LPPC increased cell cycle regulators (p53, p-p53, and p21) and decreased cell cycle-related proteins (Rb, p-Rb, CDK4, and cyclin D1), leading to cell cycle arrest at the G_0_/G_1_ phase in HCC cells. BP/LPPC induced cell apoptosis through activation of both the extrinsic (Fas-L and Caspase-8) and intrinsic (Bax and Caspase-9) apoptosis pathways and activated the caspase cascade to trigger HCC cell death. In conclusion, the LPPC complex improved the antitumor activity of BP in terms of cytotoxicity, cell cycle regulation and cell apoptosis, and BP/LPPC synergistically inhibited cell growth during combination treatment with VP-16 in HCC cells. Therefore, BP/LPPC is potentially a good candidate for clinical drug development or for use as an adjuvant for clinical drugs as a combination therapy for hepatocellular carcinoma.

## 1. Introduction

Hepatocellular carcinoma (HCC) represents the second and sixth leading cause of cancer death in men and woman worldwide, respectively. It is especially prevalent in East Asia and sub-Saharan Africa, where it is one of the leading causes of cancer-related death [1–3]. Because of the long duration of HCC, most patients are diagnosed in the intermediate or advanced stages, for which chemotherapy is the only option. However, there is a low response rate and a high rate of severe side effects for chemotherapy in HCC patients [4]. Conventional chemodrugs have high toxicity and lack selectivity between cancer cells and normal cells, and it has been reported that chemodrugs accumulate in tumor tissue at 5-10% of the dose that accumulates in normal organs [5]. Therefore, the poor accumulation of chemodrugs leads to poor prognosis, cancer recurrence, and poor survival. It is urgent that new therapeutic options with high anticancer effects and low cytotoxicity for normal cells are developed for HCC therapy.

Drug carriers, such as polymer-based liposomes, have improved the effects of drugs. These carriers protect the natural compound, decrease the drug penetration of normal organs, and increase the cytotoxicity of the drug in tumor cells [6–8]. Previous studies showed liposome-enhanced anticancer effects in colon carcinoma, osteosarcoma, pancreatic cancer, and hepatocellular carcinoma in vitro and in vivo [9–12]. Polycationic Liposome Containing PEI and Polyethylene Glycol Complex (LPPC), a novel modified liposome, has a lipid bilayer composed of DOPC and DLPC that is noncovalently modified with PEG and PEI [13]. The LPPC technology enhanced antitumor effects by triggering the rapid penetration of drugs into tumor areas to suppress tumor growth and increase drug cytotoxicity in drug-resistant cancer [14]. Additionally, the LPPC-delivery system had improved drug transport properties and therapeutic efficacy, suggesting that it is a promising new tool for cancer therapy [15–17].

Recent studies showed that n-butylidenephthalide (BP), a natural compound from *Angelica sinensis*, which is used in traditional Chinese medicine for menopausal symptoms, had dramatic antitumor effects for glioblastoma, colon cancer, lung cancer, and hepatoma [18–23]. BP induces cell cycle arrest through increases in cyclin kinase inhibitors such as p21 and p27, and it inhibits the ERK1/2 pathway to suppress tumor growth. However, BP is quickly metabolized by the liver and excreted in urine within 24 h, and the short half-life in serum of rats is approximately 12 h [20, 22, 24]. Moreover, when BP is dissolved in a water solution, the molecular structure of BP will be hydrated or oxidized, resulting in the loss of the bioactivity that is imitated for the development of clinical chemotherapy [25–28].

LPPC encapsulation of BP maintains its structural stability and enhances its antitumor effects; moreover, BP/LPPC complex carrier has a positive zeta-potential that triggers cellular uptake of drugs in glioblastoma and melanoma [28–30]. In this study, we investigated the protection and enhancement of BP-induced antitumor effects in HCC cells when BP is encapsulated in LPPC and the possible mechanisms of these effects.

## 2. Materials and Methods

### 2.1. Cell Lines and Drug Treatment

Three kinds of human hepatocellular carcinoma cells were included: HepG2, Mahlavu, and J5. Two normal cell lines were used: MDCK (canine kidney epithelial cells) and SVEC (mouse endothelia cells). All cells were obtained from the Food Industry Research and Development Institute (Hsinchu, Taiwan). The culture medium for HepG2, Mahlavu, MDCK, and SVEC cells was Dulbecco's Modified Eagle medium, and the culture medium for J5 cells was RPMI-1640. Heat-inactivated fetal bovine serum (10%; Gibco BRL, Gaithersburg, Maryland), HEPES (10 mM; Gibco), pyruvate (1 mM; Gibco), and P/S (100 units/ml Penicillin and 100 *μ*g/ml Streptomycin; Gibco) were added to the media. Those cells were subcultured with 0.25%-0.5% trypsin in EDTA solution and were cultured in growth medium in a humidified atmosphere with 5% CO_2_ at 37°C. The p53 status was wild type in HepG2 cells, but it was mutated in Mahlavu cells, as detected through a method of automated extraction of nucleic acids (AccuBioMed Co., Ltd., Taipei, Taiwan) and PCR with the Femtopath human TP53 Exon8 Primer Set (HongJing Biotech, Taipei, Taiwan).

n-Butylidenephthalide (BP) was purchased from Lancaster Synthesis Ltd. (Newgate, Morecambe, UK) and was encapsulated with LPPC (from Kuang-Wen Liao lab, National Chiao Tung University, Taiwan) according to a previously reported protocol [28]. Cells were treated with BP or BP/LPPC for various lengths of time and at various doses. Etoposide (VP-16) was purchased from Sigma-Aldrich (St. Louis, MO, USA).

### 2.2. Analysis of Cytotoxicity

Cells were incubated in each well of 96-well culture plates (5 × 10^3^ cells per well) overnight and were treated with BP/LPPC (0–100 *μ*g/ml) or BP (0–400 *μ*g/ml) for 24 and 48 h. The medium of each well was replaced with 100 *μ*l MTT solution (400 *μ*g/ml, Sigma-Aldrich) for 6–8 h incubation. The MTT solution was removed, 50 *μ*l of DMSO was added to each well to dissolve the formazan crystal, and the absorbance was measured by a microplate reader (Molecular Device/Spec384) at 550 nm. The cell viability of cells with no drug treatment was a control for 100% viability.

### 2.3. Protective Effect of BP Activity

The protective effect of BP activity via LPPC encapsulation was evaluated by the improvement in cytotoxic activity of BP incubated in different environments. BP/LPPC and nonencapsulated BP, both at concentrations of 3 mg/ml, were incubated in ddH_2_O at 4°C or protein-rich solutions (10% FBS in PBS) at 37°C for 0, 4, 8, or 24 h. HepG2 and J5 cells were treated with the incubated-BP/LPPC or BP solutions, and the IC_50_ values were calculated by MTT assay.

### 2.4. Analysis of BP Uptake

The cells were seeded at a density of 5 × 10^5^ cells per dish in 3.5 cm^2^ dishes that contained 15 mm microscope cover glasses (Assistant, Germany) and were incubated overnight. The cells were treated with BP/LPPC (50 *μ*g/ml) or BP (50 *μ*g/ml) for 0, 15, 30, 45, or 60 min. The cover glasses were taken out, and the cells were fixed with 10% formalin. The blue fluorescence of BP and cell morphology were observed under an upright fluorescence microscope (ZEISS AXioskop2) at a magnification of 400x.

HepG2 cells were incubated in 24-well culture plates (2.5 × 10^5^ cells per well) overnight and were treated with BP/LPPC (50 *μ*g/ml) or BP (50 *μ*g/ml) for 0, 15, 30, 45, or 60 min. The treated cells were collected, and phenol-chloroform extraction was performed. BP values in were determined by a fluorescence spectrophotometer (HITACHI F-4500) at 350 nm [28].

### 2.5. Determination of Endocytosis Pathway

Cells were plated in each well of 24-well culture plates (2.5 × 10^5^ cells per well) and were incubated overnight. After the medium was removed from the cells, they were pretreated for 1 h with different endocytosis inhibitors, including amiloride hydrochloride hydrate (AHH, 13.31 *μ*g/ml, Sigma-Aldrich, USA), filipin III (FIII, 1 *μ*g/ml, Sigma-Aldrich, USA), and chlorpromazine hydrochloride (CPZ, 10 *μ*g/ml, Sigma-Aldrich, USA), and then, they were treated with BP/LPPC (50 *μ*g/ml) for 0, 15, 30, 45, or 60 min. Finally, the BP value in the cells was calculated by the method described above.

### 2.6. Cell Cycle Analysis

HepG2 cells were seeded in 10 cm^2^ dishes (2 × 10^6^ cells per dish) overnight and were treated with BP/LPPC or BP. After the cells were treated, the cells were pelleted and then resuspended with 800 *μ*l PBS containing 100 *μ*l PI (400 *μ*g/ml, Sigma-Aldrich) and 100 *μ*l RNase (1 mg/ml, Sigma-Aldrich). The cells were incubated at 4°C overnight. The cell cycle was analyzed for FL2 intensity using FACScan (Beckton Dickinson, USA) and Kaluza Flow Cytometry Analysis Software (Software version 1.2, Beckman Coulter, USA).

### 2.7. TUNEL Assay

Apoptosis was detected by using the In Situ Cell Death Detection Kit, POD (Roche, Mannheim, Germany). The treated cells were fixed with 10% formalin and dried on silane-coated glass slides (MATSUNAMI, Tokyo, Japan). The cells were rehydrated with PBS, exposed to 3% H_2_O_2_ in methanol for 10 min to decrease the activity of endogenous peroxidase, and incubated with cold permeabilization solution (0.1% Triton X-100 in 0.1% sodium citrate) for 2 min. Then, the cells were incubated with TUNEL reaction mixture for 2 h at 37°C and were counterstained with PI. The cell apoptotic morphology was observed by fluorescence microscopy (ZEISS AXioskop2) at 400x magnification.

### 2.8. Western Blotting

Cell pellets were resuspended with RIPA buffer mixture solution, and the protein concentration was measured by a bicinchoninic acid (BCA) protein assay kit (Pierce, Rockford, IL, USA). Proteins (20 *μ*g) of cell lysates were separated, detected, and analyzed according to a published protocol [30]. The primary antibodies used in the western blots were anti-p53, anti-phospho-p53, anti-Rb, anti-phospho-Rb, anti-p21, anti-CKD4, anti-cyclin D1, anti-Fas-L, anti-Bax, anti-caspase 3, anti-caspase 8, and anti-caspase 9 (Santa Cruz, CA, USA) or anti-*β*-actin (iReal Biotechnology, Hsinchu, Taiwan). The relative expression of these proteins was determined by the protein expression index = (sample intensity/*β*‐actin intensity of sample)/(control intensity/*β*‐actin intensity of control).

### 2.9. Combination Effect Analysis

The combination effect analysis was designed such that HepG2 cells (5 × 10^3^ cells per well) were treated with BP/LPPC (0, 2.5, 5, 10, 20, or 40 *μ*g/ml) combined with 2.5 *μ*g/ml VP-16 or VP-16 (0, 0.625, 1.25, 2.5, 5, or 10 *μ*g/ml) combined with 15 *μ*g/ml BP/LPPC for 48 h. The cell viability was detected by MTT assay. The combination index (CI) value = [(drug A + B) IC_50_/(drug A) IC_50_] + [(drug A + B) IC_50_/(drug B) IC_50_]. The treatments were defined as having an additive effect (CI = 1), synergism (CI < 1), or antagonism (CI > 1) [31].

### 2.10. Statistical Analysis

All results are expressed as the means ± SD (standard deviation) from at least three independent experiments. Student's *t*-test or one-way ANOVA was used to analyze statistical significance. A *p* value < 0.05 was considered statistically significant.

## 3. Results

### 3.1. BP/LPPC Induced Cytotoxicity in HCC Cells

Illustration of LPPC with BP is shown in Figure 1(a). Our previous study demonstrated that the maximal encapsulation capacity of LPPC (1 mg) was ~830 *μ*g of BP [28]. The average particle size of BP/LPPC (a 3 : 10 ratio of BP and LPPC) was ~280 nm, and the zeta-potential was ~38 mV. In vitro drug release after 5-day incubation, the percentage of encapsulated BP released from BP/LPPC was ~6.5% at 4°C and ~22% at 37°C.

The growth inhibition curves of BP/LPPC and BP in HepG2 and J5 cells were measured by MTT assays (Figures 1(b) and 1(c)). The BP/LPPC group (10.46–15.50 *μ*g/ml) revealed lower IC_50_ values than the BP group (64.42–103.06 *μ*g/ml) and the BP/liposome group (111.29–154.45 *μ*g/ml) in HCC cells (Table 1). However, BP/LPPC treatment resulted in lower cytotoxicity in the normal cells (26.20–33.92 *μ*g/ml) than in the HCC cells (10.46–15.50 *μ*g/ml). The results indicated that BP/LPPC had higher cytotoxicity than BP and BP/liposome in HCC cells but lower cytotoxicity in normal cells than in HCC cells.

### 3.2. LPPC Protected BP Activity for Cytotoxicity of HCC Cells

To analyze the protection effect of LPPC encapsulation on BP activity, the drugs prepared for the BP/LPPC group (encapsulated BP) and for the BP group (nonencapsulated BP) were stored at 4°C or 37°C in different environments, and the drug preparations were incubated for 0, 4, 8, or 24 h. In Figure 2, BP/LPPC prepared in ddH_2_O solution and incubated at 4°C had higher cytotoxicity in the two HCC cell lines (IC_50_ = 12.52–12.93 *μ*g/ml, 0 h; IC_50_ = 19.17–23.83 *μ*g/ml, 24 h) than the BP prepared in the same way (IC_50_ = 50.36–97.36 *μ*g/ml, 0 h; IC_50_ = 243.20–275.08 *μ*g/ml, 24 h). In when prepared in a protein-rich medium and incubated at 37°C, BP/LPPC also showed higher cytotoxicity (IC_50_ = 17.41–18.68 *μ*g/ml, 0 h; IC_50_ = 30.69–36.00 *μ*g/ml, 24 h) than BP (IC_50_ = 47.53–95.61 *μ*g/ml, 0 h; IC_50_ = 211.40–222.94 *μ*g/ml, 24 h). The data suggest that BP was quickly losing activity after it was prepared in an aqueous solution, but LPPC encapsulation protected the cytotoxicity of BP in HCC cells.

### 3.3. LPPC Enhanced Cell Uptake of BP through Endocytosis

Due to its positive zeta-potential (~38 mV), BP/LPPC was able to induce endocytosis and enhance cell uptake in HCC cells. After the cells were treated with BP/LPPC or BP, BP uptake was determined quantitatively by measuring BP fluorescence. BP fluorescence was detected in the BP/LPPC group after 15 min of incubation and in the BP group after 60 min of incubation, indicating that LPPC encapsulation triggered a more rapid BP penetration into HepG2 cells (Figure 3(a)). However, both BP/LPPC and BP treatments resulted in slow cellular uptake of BP in MDCK cells (Figure 3(b)).

As shown in Figure 3(c), in HepG2 cells treated for 15-60 min, the values of total BP uptake in the BP/LPPC group (12.57–20.81 *μ*g) were higher than those of the BP group (1.35–8.01 *μ*g). In MDCK cells, the cellular uptake of BP after a 60 min incubation period was lower in both the BP/LPPC group (2.37–7.50 *μ*g) and the BP group (2.20–7.05 *μ*g) than in the HepG2 cells. The results revealed that LPPC encapsulation promoted the efficiency of BP uptake in HCC cells, but not in normal cells.

To investigate the cellular uptake mechanism, HepG2 cells were pretreated with endocytosis inhibitors, including AHH (micropinocytosis inhibitor), FIII (caveola-mediated endocytosis inhibitor), or CPZ (clathrin-mediated endocytosis inhibitor) [32]. Then, the cells were treated with BP/LPPC and collected, and the BP values were measured. In treatment for 15-90 min, the BP values in cells were decreased in all inhibitor groups relative to the control group (12.57–16.94 *μ*g), especially in FIII groups (9.69–15.09 *μ*g), shown in Figure 3(d). The results showed that positively charged BP/LPPC triggered cellular uptake of BP in HepG2 cells through caveola-mediated endocytosis.

### 3.4. BP/LPPC Induced Cell Cycle Arrest at the G_0_/G_1_ Phase in HepG2 Cells

HepG2 cells were treated with BP/LPPC or BP, and the cell cycle distribution was analyzed for FL2 intensity by FACScan. The results revealed that the cell cycle was arrested at the G_0_/G_1_ phase after BP/LPPC and BP treatment in HCC cells (Figures 4(a)–4(d)). The relative protein expression of cell cycle proteins in treated cells was detected by western blotting. The protein expression of cell cycle regulators (p21, p53, and p-p53) was increased, and the expression of tumor suppressor proteins (p-Rb and Rb) was decreased (Figures 4(e) and 4(f)). Additionally, cell cycle proteins CDK4 and cyclin D1 were decreased after BP/LPPC and BP treatment. Thus, BP/LPPC and BP regulated cell cycle-related protein expression and induced cell cycle arrest at the G_0_/G_1_ phase.

### 3.5. BP/LPPC Induced Extrinsic and Intrinsic Cell Apoptosis in HepG2 Cells

After BP/LPPC or BP treatment, the percentage of SubG_1_ phase was increased in time- and dose-dependent manners (Figures 5(a)–5(c)). Additionally, BP/LPPC and BP-treated cells exhibited apoptotic morphology, including chromatin condensation, DNA fragmentation, and apoptosis bodies, as detected through the TUNEL assay Figure 5(d)). The molecules of the extrinsic apoptosis pathway (Fas-L and caspase-8) and the intrinsic pathway (Bax and caspase-9) were activated after BP/LPPC and BP treatment, as observed by western blot (Figures 5(e) and 5(f)). Finally, cleaved caspase-3 turned on the caspase cascade and triggered cell death. The BP/LPPC treatment (60 *μ*g/ml) group had a higher activation effect on caspase-3, caspase-8, and caspase-9 than the BP treatment (120 *μ*g/ml) group at 6 h. The results demonstrated that BP/LPPC and BP induced cell apoptosis via activation of the extrinsic and intrinsic apoptosis pathways in HCC cells.

### 3.6. BP/LPPC Combined with VP-16 Showed a Synergistic Effect

To determine the effect of BP/LPPC combined with clinical drug etoposide (VP-16), an experiment was designed in which cells were treated with BP/LPPC (0–40 *μ*g/ml) combined with 2.5 *μ*g/ml VP-16 or with VP-16 (0–10 *μ*g/ml) combined with 15 *μ*g/ml BP/LPPC. After treatment, the groups that received BP/LPPC at doses of 0, 2.5, or 5 *μ*g/ml combined with VP-16 (2.5 *μ*g/ml) for 48 h had higher cytotoxicity (69.26%, 59.77%, or 52.92%) than the groups that received BP/LPPC only (100%, 94.27%, or 85.19%, Figure 6(a)). In addition, the cell viability was decreased in the groups that received VP-16 at doses of 0, 0.63, or 1.25 *μ*g/ml combined BP/LPPC (15 *μ*g/ml) for 48 h (52.20%, 40.34% or 37.26%) than the groups that received VP-16 only (100%, 80.82%, or 74.33%, Figure 6(b)). The combination index (CI) value was 0.52 between BP/LPPC and VP-16, suggesting that BP/LPPC combined with VP-16 synergistically inhibited the growth of HCC cells.

## 4. Discussion

HCC represents the second and sixth leading cause of cancer death in men and women in global cancer statistics 2018 for 36 cancers of 185 countries, respectively, and five-year survival rates of up to 60 to 70% can be achieved in well-selected patients [1–3]. Unfortunately, the disease is often diagnosed at the intermediate or advanced stages, for which chemotherapy is the only treatment choice. However, the therapeutic effects are comparatively poor, and patients undergo various adverse effects due to off-target effects of the chemotherapy on noncancerous organs and tissues [4]. Polymer-based liposomes improve the effects of drugs, including reducing the drug penetration of normal organs, protecting the activity of natural compounds, and increasing the cytotoxicity of drug compounds in tumor cells [6–8]. Thus, the aim of this study was to develop a novel BP-loaded Lipo-PEG-PEI complex and to characterize its pharmaceutical properties and cytotoxic activity against HCC cells in vitro.

Previous studies showed that cationic liposomes improve cellular uptake via induction of endocytosis [33, 34]. BP/LPPC complex carrier has a positive zeta-potential (~38 mV), which enhances cellular uptake of drugs in tumor cells [28–30]. In this study, the results revealed that BP/LPPC penetrated more quickly into HCC cells than nonencapsulated BP, and the increase in total BP uptake was more than 2.6-fold at 60 min. However, there was no significant difference between BP/LPPC and BP in canine kidney epithelial cells (MDCK cells). Moreover, BP/LPPC induced cell cycle arrest at the G_0_/G_1_ phase at lower a dose compared with BP. This BP/LPPC-induced cell cycle arrest was regulated by changes in p53/p21 and CDK4/cyclin D1 protein expression, and cell apoptosis was induced by the activation of extrinsic (Fas-L/Cas-8) and intrinsic (Bax/Cas-9) pathways. The results suggested that LPPC triggers cellular uptake of BP in tumor cells but not in normal cells, indicating that BP/LPPC is highly selective to tumor cells. Additionally, through the pretreatment of cells with endocytosis inhibitors, including AHH (macropinocytosis), FIII (caveola-mediated endocytosis), or CPZ (clathrin-mediated endocytosis) [32], we found that LPPC activates different endocytosis pathways, especially the caveola-mediated pathway, to increase cellular uptake of BP in HCC cells, thereby causing cell death.

Several studies have indicated that n-butylidenephthalide (BP), which is a natural compound, has an unstable structure that easily undergoes oxidation, hydration, and dimer formation, which lead to a rapid reduction in BP activity when BP is dissolved in aqueous solutions [25–28]. Our recent study showed that Polycationic Liposome Containing PEI and Polyethylene Glycol Complex (LPPC) can protect BP activity and enhance the antitumor effects of BP in glioblastoma and melanoma [28–30]. In this study, we demonstrated that LPPC protected BP activity not only in a 4°C aqueous solution but also in a 37°C protein-rich solution. LPPC enhanced the cellular uptake of BP in HCC cells, which indicates that LPPC is promising for improving the development of BP for clinical chemotherapy.

Chemotherapy treatment of HCC has high adverse effects after the therapeutic course due to low selection between tumor cells and normal cells [4, 5]. In this study, the results indicated that the speed of cellular uptake of BP was slower in normal cells than in HCC cells and that the total amount of BP taken up was lower in normal cells than in HCC cells. Additionally, BP/LPPC had lower cytotoxicity in normal cells compared with HCC cells, suggesting that BP/LPPC uptake and cytotoxic effects were more specific to HCC cells than to normal cells. However, the clinical drug VP-16 showed lower selection between normal cells and HCC cells. Moreover, BP/LPPC combined with VP-16 synergistically inhibited the growth of HCC cells, suggesting that VP-16 combined with BP/LPPC could decrease the usage dose of VP-16 to moderate its adverse effects. Therefore, BP/LPPC may be developed as a chemotherapeutic drug combined with VP-16 or alone to reduce the occurrence of adverse events in HCC patients during chemotherapy.

## 5. Conclusion

LPPC encapsulation improves cellular uptake of BP, protects BP activity, and enhances BP-induced cytotoxicity in HCC cells. Additionally, BP/LPPC combined with VP-16 showed synergistic growth inhibition in HCC cells. As part of its antitumor mechanism, BP/LPPC induces cell cycle arrest at the G_0_/G_1_ phase by regulating p53/p21 and CDK4/cyclin D1 protein expression and by activating both the intrinsic and extrinsic apoptotic pathways to induce cell death. Therefore, BP/LPPC has high potential to be developed as a clinical chemodrug for hepatocellular carcinoma.

## Figures and Tables

**Figure 1:** BP/LPPC induced cytotoxicity in HCC cells. (a) Illustration of LPPC with BP. The BP was loaded in lipid layer of LPPC. (b) HepG2 and (c) J5 cells were treated with BP/LPPC (0–100 *μ*g/ml) or BP (0–400 *μ*g/ml) for 24 or 48 h. The percentage of cell viability was measured by the MTT assay.

**Figure 2:** LPPC encapsulation protected BP activity and cytotoxicity. BP/LPPC and BP stored in ddH_2_O at 4°C or in protein-rich solution (10% FBS in PBS) at 37°C for 0, 4, 8 or 24 h. (a) HepG2 and (b) J5 cells were treated with incubated-BP/LPPC or BP for 24 h, and the IC_50_ was calculated by using the MTT assay. ∗: Significant difference compared with 0 h in the ddH_2_O group (*p* <0.05). #: Significant difference compared with 0 h in the protein-rich solution group (*p* <0.05).

**Figure 3:** Promotion of BP uptake into HCC cells by LPPC encapsulation. To analyze BP uptake in tumor or normal cells, (a) HepG2 and (b) MDCK cells were incubated with 50 *μ*g/ml BP/LPPC or BP, and BP uptake was observed on an upright fluorescence microscope (blue fluorescence). DIC, differential interference contrast. (c) The value of BP uptake in cells was quantitated by detection of fluorescence in a spectrophotometer. ∗: Significant difference between BP/LPPC and BP group (*p* <0.05). (d) HepG2 cells were pretreated with endocytosis inhibitors (AHH, FIII or CPZ) for 1 h and were then treated with 50 *μ*g/ml BP/LPPC. BP values in cells were calculated. a: Significant difference in the AHH group compared with the no inhibitor group (*p* <0.05). b: Significant difference in the FIII group compared with the no inhibitor group (*p* <0.05). c: Significant difference in the CPZ group compared with the no inhibitor group (*p* <0.05).

**Figure 4:** BP/LPPC and BP induced cell cycle arrest at the G_0_/G_1_ phase in HCC cells. (a–d) The HepG2 cells were treated with BP/LPPC or BP, and then, cell cycle analysis for FL2 intensity was measured by FACScan. Each column showed mean ± SD. ∗: Indicates a significant increase compared with control (*p* <0.05). #: Indicates a significant decrease compared with control (*p* <0.05). (e, f) Cell cycle-related protein expression was detected by using western blotting.

**Figure 5:** BP/LPPC activated caspase cascade to trigger cell apoptosis in HCC cells. (a–c) HepG2 cells were treated with BP/LPPC or BP, and the percentage of SubG_1_ phase was measured by using FACScan. ∗: Indicates a significant increase compared with control (*p* <0.05). (d) Cell apoptosis in BP/LPPC and BP-treated cells were determined by using TUNEL assay, and apoptosis morphology (I, chromatin condensation; II, DNA fragmentation; III, apoptotic body) was observed under fluorescence microscopy (400×). (e, f) Apoptosis-associated protein expression was detected by using western blotting.

**Figure 6:** BP/LPPC combined with VP-16 synergistically inhibited the growth of HCC cells. (a) HepG2 cells were treated with BP/LPPC (0, 2.5, 5, 10, 20 or 40 *μ*g/ml) combined with VP-16 (2.5 *μ*g/ml) for 48 h. (b) HepG2 cells were treated with VP-16 (0, 0.63, 1.25, 2.5, 5 or 10 *μ*g/ml) combined with BP/LPPC (15 *μ*g/ml) for 48 h. ∗: Represents a significant difference compared with 0 h in the combination group (*p* <0.05).

**Table 1:** The IC_50_ values of BP and BP/LPPC against HCC cell lines.

Cell line	BP (A)	BP/LPPC (B)	BP/Lipo	VP-16	Fold (*A*/*B*)
*HCC cells*					
HepG2	64.42 ± 2.50	11.12 ± 3.00^a,b,c^	154.45 ± 5.79	60.34 ± 1.00	5.79
Mahlavu	103.06 ± 3.54	15.50 ± 2.84^a,b^	119.78 ± 0.42	ND	6.65
J5	71.33 ± 2.08	10.46 ± 1.91^a,b,c^	111.29 ± 2.27	137.79 ± 1.54	6.82
*Normal cells*					
SVEC	107.24 ± 2.25	26.20 ± 0.24^a,c^	ND	3.12 ± 3.02	4.09
MDCK	128.30 ± 1.96	33.92 ± 1.75^a,b^	171.01 ± 2.85	35.15 ± 1.59	3.78

The IC_50_ values revealed the concentration that results in a 50% decrease of cell viability. Values are the mean ± SD (*μ*g/ml) at 24 h. The fold (*A*/*B*) was the IC_50_ value ratio of BP and BP/LPPC. BP/Lipo: BP/liposome; ND: nondetection. ^a^Significant difference in BP/LPPC treatment compared with BP treatment (*p* < 0.05). ^b^Significant difference in BP/LPPC treatment compared with BP/Lipo treatment (*p* < 0.05). ^c^Significant difference in BP/LPPC treatment compared with VP-16 treatment (*p* < 0.05).

## Data Availability

All data generated or analyzed during this study are included in this article.
